The article "Unsupervised Clustering Reveals Sarcoidosis Phenotypes Marked by a Reduction in Lymphocytes Relate to Increased Inflammatory Activity on 18FDG-PET/CT" was published in 2021. Journal: Front Med (Lausanne).

# Unsupervised Clustering Reveals Sarcoidosis Phenotypes Marked by a Reduction in Lymphocytes Relate to Increased Inflammatory Activity on 18FDG-PET/CT

**DOI:** 10.3389/fmed.2021.595077

**Published:** 2021-02-24

**Authors:** Christen Vagts, Christian Ascoli, Dustin R. Fraidenburg, Robert P. Baughman, Yue Huang, Russell Edafetanure-Ibeh, Samreen Ahmed, Benjamin Levin, Yang Lu, David L. Perkins, Patricia W. Finn, Nadera J. Sweiss

**Affiliations:** ^1^Division of Pulmonary, Critical Care, Sleep, and Allergy, Department of Medicine, University of Illinois at Chicago, Chicago, IL, United States; ^2^Department of Internal Medicine, University of Cincinnati Medical Center, Cincinnati, OH, United States; ^3^Division of Rheumatology, Department of Medicine, University of Illinois at Chicago, Chicago, IL, United States; ^4^Division of Cardiology, Department of Medicine, College of Medicine, University of Illinois at Chicago, Chicago, IL, United States; ^5^Jesse Brown VA Medical Center, Chicago, IL, United States; ^6^Division of Diagnostic Imaging, Department of Nuclear Medicine, The University of Texas MD Anderson Cancer Center, Houston, TX, United States; ^7^Division of Nephrology, Department of Medicine, University of Illinois at Chicago, Chicago, IL, United States

**Keywords:** sarcoidosis, lymphopenia, 18FDG-PET/CT, immunopathogenesis, cluster analysis, phenotype

## Abstract

**Introduction:** Sarcoidosis is a T-helper cell mediated disease characterized by granulomatous inflammation. We posited that unsupervised clustering of various features in sarcoidosis would establish phenotypes associated with inflammatory activity measured by 18FDG-PET/CT. Our goal was to identify unique features capable of distinguishing clusters and subsequently examine the relationship with FDG avidity to substantiate their potential use as markers for sarcoidosis inflammation.

**Methods:** We performed a retrospective study of a diverse, but primarily African American, cohort of 58 subjects with biopsy proven sarcoidosis followed at the University of Illinois Bernie Mac Sarcoidosis Center and Center for Lung Health who underwent 18FDG-PET/CT scan. Demographic, therapeutic, radiographic, and laboratory data were utilized in unsupervised cluster analysis to identify sarcoidosis phenotypes. The association between clusters, their defining features, and quantitative measurements on 18FDG-PET/CT was determined. The relevance of these features as markers of 18FDG-PET/CT inflammatory activity was also investigated.

**Results:** Clustering determined three distinct phenotypes: (1) a predominantly African American cluster with chronic, quiescent disease, (2) a predominantly African American cluster with elevated conventional inflammatory markers, advanced pulmonary disease and extrathoracic involvement, and (3) a predominantly Caucasian cluster characterized by reduced lymphocyte counts and acute disease. In contrast to the chronic quiescent cluster, Clusters 2 and 3 were defined by significantly greater FDG avidity on 18FDG-PET/CT. Despite similarly increased inflammatory activity on 18FDG-PET/CT, Clusters 2, and 3 differed with regards to extrathoracic FDG avidity and circulating lymphocyte profiles, specifically CD4+ T-cells. Notably, absolute lymphocyte counts and CD4+ T-cell counts were found to predict 18FDG-PET/CT inflammatory activity by receiver operating curve analysis with a 69.2 and 73.42% area under the curve, respectively.

**Conclusions:** Utilizing cluster analysis, three distinct phenotypes of sarcoidosis were identified with significant variation in race, disease chronicity, and serologic markers of inflammation. These phenotypes displayed varying levels of circulating inflammatory cells. Additionally, reduction in lymphocytes, specifically CD4+ T-cells, was significantly related to activity on 18FDG-PET/CT. Though future studies are warranted, these findings suggest that peripheral lymphocyte counts may be considered a determinant of sarcoidosis phenotypes and an indicator of active inflammation on 18FDG-PET/CT.

## Introduction

Sarcoidosis is a heterogeneous multisystem disease characterized by granulomatous inflammation. While sarcoidosis affects a variety of races, African American women have the highest prevalence of disease and new cases most commonly are diagnosed in the 4th and 5th decades of life (1). Sarcoidosis has been characterized as a T-helper cell mediated disease (2). The ACCESS trial identified genetic risk factors for sarcoidosis development in various races, and some genes were linked to immune dysregulation and decreased lymphocytes in a Caucasian subset of this cohort (3, 4). Moreover, despite the lack of sarcoidosis specific thresholds, absolute lymphocyte counts ≤ 1.5 kcells/μL have been associated with disease activity and progression (5, 6). Peripheral depletion of CD4+, CD8+, and CD19+ T-cells has also been shown to be a characteristic of patients with severe sarcoidosis (7). Furthermore, lymphocyte gene expression is decreased in patients with severe disease and CD4+ T-cell exhaustion has been described as a manifestation of progressive disease (8, 9). Thus, further characterization of lymphopenia, as it relates to disease pathogenesis and inflammation, merits investigation within specific phenotypes of sarcoidosis.

Given the heterogeneous nature of sarcoidosis, establishing disease phenotypes is critical to identify common pathways that may further shed light on disease etiology and pathogenesis. Existing phenotypes in sarcoidosis have focused on subject and disease characteristics, to include radiographic staging, organ involvement, disease acuity, and need for treatment (10–12). Even though useful clinical tools have been proposed, the classification criteria for various clinical phenotypes of sarcoidosis are not well-standardized and criteria for research purposes are lacking (13). Cluster analysis techniques have been utilized in diseases that are difficult to classify, including other autoimmune and pulmonary diseases, and have yielded novel insights (14–18). To this end, a recent report utilized cluster analysis of a large predominantly Caucasian sarcoidosis cohort and identified 6 subsets of subjects that better predicted disease progression than classical analysis (19). A second study utilized a supervised hierarchical cluster analysis to identify phenotypes of sarcoidosis based on 18FDG-PET/CT (PET scan) uptake. Cluster and PET scan analyses provided a meticulous evaluation of organ involvement and a more precise evaluation of the extent of disease compared to traditional assessment (20). Cluster analysis has therefore proven helpful at identifying similarities of disease beyond conventional classification schemes which may have implications for treatment and prognostication.

PET scan is an emerging tool for assessing inflammation in sarcoidosis as well as other inflammatory and autoimmune disorders (21, 22). Uptake on PET scan, commonly defined as SUV >2.5, has been consistently associated with disease activity as well as pulmonary function in patients with sarcoidosis (23–25). The sensitivity of PET scan in identifying active inflammation ranges 89–100% and is overall higher when compared to traditional biomarkers (24). PET scan use has been evaluated in both acute and chronic disease, is superior at detecting ongoing inflammation in persistent disease, and shows promise in guiding treatment and prognosis (26–28). We posited the usefulness of PET scan as a tool in the absence of a biomarker specific enough to monitor inflammation in sarcoidosis (29). ATS guidelines support use of PET scan to assess extracardiac sarcoidosis, albeit with low quality of evidence, suggesting further research is needed to develop a disease specific biomarker with adequate sensitivity to serve as a more cost-effective assessment strategy (30).

Our goal was to identify unique phenotypes of sarcoidosis using an unsupervised cluster analysis in subjects with biopsy proven sarcoidosis in order to establish the relationship between these phenotypes and inflammatory activity, as measured by serologic markers of inflammation and avidity on 18FDG-PET/CT scan. Our postulate was that a parsimonious set of demographic features along with clinically relevant therapeutic, radiographic, and laboratory features would identify subgroups of subjects with sarcoidosis at risk of active disease characterized by high levels of inflammation.

## Methods

### Subject Selection

Study approval was obtained through the University of Illinois at Chicago (UIC) institutional review board. Adult subjects 18 years of age and older followed in the Bernie Mac Sarcoidosis Translational Advanced Research (STAR) Center at UIC with a history and tissue biopsy consistent with sarcoidosis, in accordance with ATS/ERS/WASOG criteria, were included (31). All subjects underwent a skull to thigh PET scan to evaluate clinically suspected metabolically active intrathoracic sarcoidosis, between December 2014 and June 2019. Subjects who had comorbid inflammatory disease that may result in increased metabolic activity on PET scan, including malignancy, connective tissue or autoimmune disease, or active infection were excluded. Subjects who did not have sufficient laboratory data available within 180 days prior or 30 days after the PET scan was completed were also excluded.

### Data Collection

The electronic medical record was retrospectively reviewed to collect variables regarding subject demographics as well as clinically relevant therapeutic, radiographic, and laboratory data. In addition to sex and self-reported race, subject demographics included age, body mass index (BMI), and smoking status at time of PET scan. Time from diagnosis to PET scan was measured from the time of biopsy. Treatment at the time of PET scan was also abstracted from medical records and categorized into the following regimens (A) naïve or local treatment, (B) systemic corticosteroids, (C) non-steroidal immune modulator, (D) combination therapy with steroids, (E) combination therapy without steroids. Laboratory values obtained within 180 days prior to or 30 days after PET scan included complete blood counts, lymphocyte subsets, serologic markers of inflammation (ESR, CRP), and markers of extrathoracic organ involvement (complete metabolic panels and vitamin D levels). ACE levels at any point prior to the PET scan were also included (Supplementary Data Sheet 1).

### PET Scan Interpretation

All 18FDG-PET/CT examinations at UIC were performed on a GE Discovery 690 FDG PET/CT scanner (GE Medical Systems, Milwaukee, WI). Dedicated PET scans from the skull base to the upper thighs were obtained 60–90 min after intravenous injection of 0.370–0.481 GBq of FDG. Image acquisition was performed using non-cardiac-gated technique with PET parameters as follows: 2 min/bed for the non-cardiac fields and 10 min/bed for fields covering the heart. Image acquisition was performed using non-cardiac-gated technique. CT scan was used for attenuation correction and parameters were as follows: 120 kV, 120 mAs, pitch 0.813, 16 × 1.5-mm collimation, slice thickness of 3 mm with an increment of 1.5 mm.

Utilizing the LIFEx radiomics software, assessment of individual PET scans in DICOM format was performed to standardize and extract functional parameter measurements in order to quantitate the burden of 18FDG-avid areas per subject with the “total metabolic tumor volume (MTV) protocol” (32). First, the maximum standardized uptake volume (SUV_Max_) as well as the mean-SUV uptake in the liver were measured and together used to calculate the SUV_Background_-to-SUV_Max_ ratio (SUV ratio). Liver mean-SUV uptake was calculated using a volume-of-interest of 3cm^3^ from the subject's right hepatic lobe. SUV ratio, shown to be a reliable measure for prognostication and treatment response, and not SUV_Max_, was utilized to minimize observer variability and standardize PET scan acquisition and reconstruction protocols (33–36). To maximize specificity of identifying a positive PET scan, lesions with a SUV ratio ≥ 2 were considered positive for inflammatory activity related to sarcoidosis, whereas those with a SUV ratio <2 were regarded as negative. This approach is similar to the use of PET scan to assess chemotherapy response in various lymphomas (35). Total Metabolic Volume (TMV), a measure of the volume of increased FDG activity in milliliters, and Total Lesion Glycolysis (TLG), the product of mean-SUV uptake with the volume of uptake, were then measured as they may better reflect overall inflammatory activity and measurement partitioned into intra- and extrathoracic compartments. Lesions included in these calculations required a minimum SUV ratio of 2, as previously noted, as well as and an SUV >40% of the SUV_Max_. These thresholds were extrapolated for use in this study as they have been shown to improve accuracy of the metabolic tumor volume measurement in various malignancies (37–39). Activity captured by the LIFEx software was then corroborated with the original radiographic interpretation of the PET scan.

### Statistical Analysis

All statistical analyses were performed with the R Statistical Environment (version 3.5.0) (40). A total of 22 subject phenotypic variables comprised of demographic, therapeutic, radiographic, and laboratory data abstracted from the electronic medical records were input as clustering features into the Modha-Spangler algorithm for mixed categorical (Table 1) and continuous (Figure 1) data in the *kamila* R-package to establish unsupervised sarcoidosis clusters. This algorithm seeks to effectively balance the contribution of continuous and categorical variables in an unsupervised fashion. In doing so, it adaptively selects the relative weight that simultaneously minimizes the within-cluster dispersion and maximizes the between-cluster dispersion for both the continuous and categorical variables (41). The Modha-Spangler framework was utilized to optimize the k-medoids algorithm PAM (partitioning around the medoids) using Gower's distance with default parameters and an optimal weight of 0.8182 by a brute-force search strategy (42). Determination of the ideal number of clusters by average silhouette width was performed utilizing the *pamk* function with criterion specifying a “krange” of 3–6 clusters given cohort heterogeneity and sample size (43).

**Table 1:** Baseline categorical parameters utilized as clustering features of the UIC-Sarcoidosis cohort (*n* = 58).

**Categorical parameters in clustering**		**Frequency (%)**
Race	Caucasian	23 (39.66)
	African American	35 (60.34)
Sex	Male	21 (36.21)
	Female	36 (63.79)
Age	30–39 years	12 (20.69)
	40–49 years	18 (31.03)
	50–59 years	22 (37.93)
	60–69 years	6 (10.35)
Body Mass Index	Normal	11 (18.97)
	Overweight	10 (17.24)
	Class 1 Obesity	11 (18.97)
	Class 2 Obesity	16 (27.59)
	Class 3 Obesity	10 (17.24)
Smoking history	Never	28 (48.28)
	Former	24 (41.38)
	Current	6 (10.34)
Time from diagnosis to 18FDG-PET/CT	Quartile 1	17 (29.31)
	Quartile 2	14 (24.14)
	Quartile 3	13 (22.41)
	Quartile 4	14 (24.14)
Lung parenchyma on CT Chest (at 18FDG-PET/CT)	Normal	21 (36.84)
	Lung Nodules	16 (28.07)
	Consolidation/GGO	8 (14.04)
	Advanced	12 (21.05)
Treatment	A	15 (25.86)
	B	15 (25.86)
	C	6 (12.07)
	D	17 (29.31)
	E	4 (6.89)
Angiotensin converting enzyme level (Ever Elevated)	No	38 (65.52)
	Yes	20 (34.49)

*Prevalence of individual parameters is depicted as frequencies and percentages. 18FDG-PET/CT, positron emission tomography with 2-deoxy-2-fluorine-18-fluoro-D-glucose with integrated computed tomography; CT, computed tomography; GGO, ground glass opacities. Time from diagnosis to 18FDG-PET/CT ranged from 0 to 27 years and quartile distribution was as follows: 1 = 0–3 years; 2 = 4–6 years; 3 = 6–10 years; 4 ≥ 11 years. Treatment regimens at time of 18FDG-PET/CT: A = naïve or local therapy; B = systemic corticosteroid alone; C = non-steroidal immune modulator alone; D = combination therapy with corticosteroid; E = combination therapy without corticosteroid*.

**Figure 1:** Box and whisker plots demonstrating baseline laboratory parameters utilized as clustering features of the UIC-Sarcoidosis cohort (*n* = 58). Values are depicted as median and interquartile ranges for each individual parameter.

Clustering features utilized in the algorithm were tested for significant differences between clusters with χ^2^-test of independence for categorical data or via Kruskal-Wallis one-way analysis of variance for continuous data *(p* ≤ 0.05 were considered statistically significant). *Post-hoc* analysis with Benjamini-Hochberg (BH) adjustment to account for the multiplicity problem that occurs with multiple comparisons was performed using Fisher's exact test for χ^2^-tests or Dunn's test for Kruskal-Wallis tests and an adjusted *p* < 0.1 was pre-specified as significant. Correlations for continuous data were performed utilizing Spearman's rank correlation coefficient and considered significant if *p* ≤ 0.05. To further investigate the probability of PET-positivity based on cluster membership a logistic regression model was constructed and odds ratios calculated.

Receiver operator characteristic (ROC) analysis with 1,000 stratified bootstrap replicates and 95% confidence intervals was performed on the cohort using the *pROC* R-package to calculate the predictive accuracy of specific cell counts with regards to determining sarcoidosis inflammatory activity on PET scan. Threshold values for specific cell counts were determined utilizing the *pROC* package's *coords* function, and the optimal numerical threshold for each cell type was calculated by maximizing sensitivities and specificities as determined by Youden's J statistic (Youden's index) (44).

## Results

There were 58 subjects identified who had a PET scan and laboratory values within the time constraints. Biopsies were predominantly obtained from lung (44.8%), lymph node (32.8%), and liver (8.6%) tissue. Thirty-five (60.34%) subjects were African American and 36 (63.79%) were women; however, the proportion of men and women within African American subjects was comparable to that of Caucasians in our cohort (χ^2^-test *p* = 0.3503). Most subjects were between 50 and 59 years of age (37.93%), though 31.03% were between 40 and 49 years and 20.69% were between age 30 and 39. There were no subjects under age 30. Time from diagnosis to PET scan, ranging from 0 to 27 years, was utilized to assess disease chronicity and distributed into quartiles. In total, 29.31% of subjects were included in quartile 1 (0–3 years), 24.14% in quartile 2 (3–6 years), 22.41% in quartile 3 (7–10 years), and 24.14% in quartile 4 (≥11 years). The most common treatment regimen was combination therapy with corticosteroid (regimen D; 17 of 58, 29.31%), though 25.86% of subjects were on corticosteroids alone (regimen B) and another 25.86% of subjects were treatment naïve (regimen A). Though there was variability in treatment regimens between subjects, individual doses and medications remained stable within the study period for each subject. Other variables, to include BMI, smoking history, lung parenchyma characteristics, and treatment are outlined in Table 1. Laboratory values utilized in clustering are summarized in Figure 1. Absolute neutrophil values in the cohort were normal while the median absolute lymphocyte count was 1.5 kcells/μL (interquartile range from 1.0 to 2.1 kcells/μL) which coincides with previously described lymphopenia defining thresholds in the general population and sarcoidosis (5, 6, 45, 46). Absolute neutrophil counts were found to be affected by treatment regimen (KW-test *p* = 0.0255); however, upon adjustment for multiple comparisons this difference was found to be specific for subjects on regimen B when compared to those on regimen A (median 5.5 vs. 3.1 kcells/μL, respectively; Dunn's test *p* = 0.0362). In contrast, subjects who were treatment naïve had a comparable prevalence of lymphocyte reduction (≤1.5 kcells/μL) to those on treatment (53.33 vs. 53.49%, respectively; χ^2^-test *p* = 0.9917). Multivariate regression analysis was performed to further assess the relationship between inflammatory cells and variables considered likely to alter their quantity (sex, race, age, BMI, smoking history, chronicity of disease, and treatment regimen) and did not identify significant associations (*p* > 0.05). Otherwise, serologic markers of inflammation were mostly within the standard reference ranges with few outliers.

Using 22 independent variables as described in Table 1, Figure 1, 3 clusters were identified (Figure 2). Characteristics of each cluster are listed in Table 2. Significant features that defined clusters included race, disease acuity, treatment, lung parenchyma, various laboratory values reflecting extrathoracic organ involvement, and serologic markers of inflammation. Cluster 1 and 2 consisted mostly of African American subjects (70.83 and 86.67%, respectively) while only 26.32% of subjects in Cluster 3 were African American (KW-test *p* = 0.0007). Subjects in Clusters 1 and 2 were mostly women (75.00 and 73.33%, respectively) while most subjects in Cluster 3 were men (57.9%); however, despite differences only a trend toward significance was noted (KW-test *p* = 0.0560). Cluster 1 had a considerably high number of subjects with PET scans performed ≥ 11 years from diagnosis and less subjects with acute disease (4.00%), while 78.94% of subjects in Cluster 3 were considered to have acute disease (KW-test *p* = 0.0004). Cluster 1 also consisted of more subjects with normal lung parenchyma on CT portion of the PET scan (77.78%) while Cluster 2 had more advanced disease (46.67%), reflected by moderate-severe emphysema and extensive fibrosis, and Cluster 3 had more lung nodules (36.85%) and either consolidation or ground glass opacities (36.84%). Cluster 1 included more treatment-naïve subjects whereas Cluster 3 had the most subjects on corticosteroid monotherapy (regimen B). Rate of any corticosteroid use (monotherapy or in combination) was highest in Cluster 2, and although a trend indicating possible difference in corticosteroid use was noted, statistical significance was not reached (χ^2^-test *p* = *0.0633)*. Cluster 2 also had more variation in laboratory values suggestive of extrathoracic organ involvement than Clusters 1 and 3, as evidenced by more elevated alkaline phosphatase (median 117 U/L, range 65.0–196.0 U/L; KW-test *p* = 0.0010), aspartate aminotransferase (median 30 U/L, range 25.0–51.5 U/L; KW-test *p* = 0.0021), and protein gap (median 3.3 g/dL, range 3.1–3.9 g/dL; KW-test *p* = 0.0131). There was no significant difference in kidney function between clusters, though there was a trend toward lower GFR in Clusters 2 and 3 than Cluster 1(KW-test *p* = 0.0853). Cluster 2 also had more subjects with abnormal serologic markers of inflammation, which included more subjects with a historically elevated ACE level (73.3%; χ^2^-test *p* = 0.0010) and a decreased 25-OH Vitamin D (median value 15.0 ng/mL; KW-test *p* = 0.0213). Variations in circulating inflammatory cells were evaluated across clusters with significant differences found in absolute neutrophil and absolute lymphocyte counts (Figure 3). In general, Cluster 1 had less abnormalities in inflammatory cell counts. Subjects in Cluster 3 had significantly higher absolute neutrophils than Cluster 1 but were not statistically different from Cluster 2 (KW-test *p* = 0.0181, median values 5.5, 3.8, and 5.2 kcells/μL, respectively). Subjects in Cluster 3 also had significantly lower absolute lymphocytes than Cluster 1 but were comparable to Cluster 2 (KW-test *p* = 0.0253, median values 1.0, 1.7, and 1.4 kcells/μL, respectively). In total, 68.42% (13/19) of subjects in Cluster 3 were found to have absolute lymphocyte counts ≤ 1.5 kcells/μL and among these 76.92% (10/13) had more evident reductions with counts ≤ 1.0 kcells/μL. Whereas, in Cluster 2, a smaller proportion of subjects (10/15) had absolute lymphocyte counts ≤ 1.5 kcells/μL of which only 30% (3/10) were found to have counts ≤ 1.0 kcells/μL. Ultimately, comparison of clusters allowed the identification of 3 phenotypic clusters: (1) a more chronic, quiescent cluster, (2) an inflammatory extrathoracic cluster with advanced pulmonary disease, and (3) a cluster with acute disease and markedly reduced lymphocyte counts.

**Figure 2:** Scatterplot visualization of the UIC-Sarcoidosis cohort over 2 dimensions utilizing the t-stochastic neighbor embedding (t-SNE) dimension reduction algorithm. The first and second dimensions are represented by the x-axis and y-axis, respectively. Points on the scatterplot represent individual subjects in the UIC-Sarcoidosis cohort and the distance between points is indicative of dissimilarity between subjects. Colors represent clusters identified by the Modha-Spangler algorithm utilizing partitioning around medoids with Gower's distance for base clustering of mixed data. Overall, Cluster 1 was identified as the largest cluster and comprised 41.38% of the cohort (24/58 subjects). Cluster 2 and 3 represented 25.86% (15/58) and 32.76% (19/58) of the cohort, respectively.

**Table 2:** Characteristics of UIC-Sarcoidosis cohort clusters.

**Cluster characteristics**		**Cluster 1**	**Cluster 2**	**Cluster 3**	***P*-value**
Race	Caucasian	7	2	14	0.0007 (β, γ)
	African American	17	13	5	
Sex	Male	6	4	11	0.056 (t)
	Female	18	11	8	
Age	30–39 years	3	2	7	NS
	40–49 years	7	5	6	
	50–59 years	12	7	3	
	60–69 years	2	1	3	
Body Mass Index	Normal	3	2	6	NS
	Overweight	5	3	2	
	Class 1 Obesity	2	6	3	
	Class 2 Obesity	10	2	4	
	Class 3 Obesity	4	2	4	
Smoking history	Never	12	7	9	NS
	Former	11	5	8	
	Current	1	3	2	
Time from diagnosis to 18FDG-PET/CT	Quartile 1	1	4	12	0.0004 (α, β)
	Quartile 2	9	2	3	
	Quartile 3	4	6	3	
	Quartile 4	10	3	1	
Lung parenchyma on CT Chest (at 18FDG-PET/CT)	Normal	14	2	6	0.0010 (α, β, γ)
	Lung nodules	4	5	7	
	Consolidation/GGO	1	1	6	
	Advanced	5	7	0	
Treatment	A	9	2	4	0.0434 (α, β)
	B	2	4	9	
	C	5	0	2	
	D	7	7	3	
	E	1	2	1	
Angiotensin converting enzyme level (Ever Elevated)	No	18	4	16	0.0010 (α, γ)
	Yes	6	11	3	
Estimated GFR (mL/min)	Median (25th-75th Percentile)	87.45 (78.0–96.4)	75.7 (68.3–82.6)	74.7 (67.4–92.9)	0.0853 (t)
Alkaline phosphatase (U/L)		76 (66.0–108.5)	117 (65.0–196.0)	58 (48.5–65.5)	0.0010 (β,γ)
Alanine aminotransferase (U/L)		23.5 (17.0–31.0)	31 (21.5–54.5)	23 (18.0–35.0)	0.0683 (t)
Aspartate aminotransferase (U/L)		26.5 (20.8–30.0)	30 (25.0–51.5)	19 (15.5–25.0)	0.0021 (β,γ)
Protein Gap (g/dL)		3 (2.7–3.5)	3.3 (3.1–3.9)	3 (2.4–3.1)	0.0131 (α,γ)
Calcium (mg/dL)		9.5 (9.3–9.8)	9.5 (9.3–9.7)	9.7 (9.4–9.8)	NS
25-Hydroxyvitamin D (ng/mL)		25 (17.8–37.5)	15 (11.5–22.0)	20 (16.0–31.0)	0.0213 (α,γ)
1, 25-Dihydroxyvitamin D (pg/mL)		57.1 (48.7–72.2)	54.8 (46.5–61.8)	52.5 (39.2–77.4)	NS
C-Reactive protein (mg/L)		0.7 (0.5–1.0)	1.1 (0.6–2.4)	06 (0.5–0.95)	NS
Erythrocyte sedimentation rate (mm/hr)		15.5 (11.8–22.8)	40 (31.0–44.5)	14 (7.5–16.0)	<0.0001 (α,β,γ)

*Numeric values for categorical variables denote frequencies and percentages. Data for continuous variables are shown as median and interquartile ranges. Comparison of features between clusters was performed utilizing χ^2^-test of independence for categorical and Kruskal-Wallis test for continuous variables. A p < 0.05 was considered significant. Post-hoc analysis with Benjamini-Hochberg (BH) adjustment for multiple comparisons was performed with Fisher's exact test for χ^2^-tests and Dunn's test for Kruskal-Wallis tests. α, β, γ denote BH-adjusted p < 0.1; α, comparison between Cluster 1 and Cluster 2; β, comparison between Cluster 1 and Cluster 3 and γ, comparison between Cluster 2 and Cluster 3. Quartiles and treatment regimens as per Table 1. NS, non-significant; t, trend*.

**Figure 3:** Box and whisker plots demonstrating median and interquartile ranges (kcells/μL) of circulating inflammatory cells in the UIC-Sarcoidosis cohort clusters. Comparisons between clusters with Kruskal-Wallis tests were performed and, if significant (*p* < 0.05), were followed by *post-hoc* analysis with Dunn's test and Benjamini-Hochberg (BH) adjustment for multiple comparisons. Kruskal-Wallis test significance is displayed in the corresponding panel and significance of Dunn's test, denoted with an asterisk (*), is displayed above the brackets linking respective box and whisker plots. Specifically, neutrophils **(A)** were found significantly elevated in Cluster 3 compared to Cluster 1 (BH-adjusted *p* = 0.0141). Conversely, lymphocytes **(B)** were found significantly reduced in Cluster 3 compared to Cluster 1 (BH-adjusted *p* = 0.0207). Neutrophil and lymphocyte counts between Cluster 1 and Cluster 2 and between Cluster 2 and Cluster 3 were comparable. Monocytes **(C)** did not show any significant differences between clusters. NS, non-significant.

With the significant differences observed in absolute lymphocyte counts between clusters, associations between cluster and the CD4+ T-cell lymphocyte subset were further evaluated (Figure 4). CD4+ T-cells correlated with absolute lymphocytes across the UIC-Sarcoidosis cohort (Spearman's rho = 0.8329, *p* < 0.0001). Between the clusters however, subjects in Cluster 3 had significantly lower CD4+ T-cells than subjects in both the chronic cluster (Cluster 1) and inflammatory extrathoracic-advanced cluster (Cluster 2), (KW-Test *p* = 0.0008, median values 421, 818, and 483 cells/μL, respectively). Interestingly, CD4+ T-cell counts in both Clusters 2 and 3 were found to be decreased in relation to reference ranges in the healthy population and sarcoidosis (7, 47, 48). CD4+ T-cells did not vary significantly between the chronic and advanced phenotypes.

**Figure 4:** Scatterplot in **(A)** demonstrates the strong direct relationship (Spearman's correlation coefficient; rho = 0.8329, *p* < 0.001) that is observed between absolute lymphocyte counts (kcells/μL) and absolute CD4+ T-cells (cells/μL). Box and whisker plots in **(B)** highlight the differences in absolute CD4+ T-cells (cells/μL) that are observed between clusters. A significant association was identified by Kruskal-Wallis test between clusters and absolute CD4+ T-cells (*p* = 0.0008). *Post-hoc* analysis with Dunn's test demonstrated significantly reduced absolute CD4+ T-cell counts, denoted with an asterisk (*), in Cluster 3 compared to Clusters 1 and 2 (BH-adjusted *p* = 0.0005 and 0.0929, respectively). No difference (NS) in absolute CD4+ T-cell counts was observed between Clusters 1 and 2.

With phenotypes supporting variable chronicity, disease location, and levels of inflammation, we proceeded to evaluate the association of these phenotypes with PET scan activity. Figure 5 describes the differences in SUV ratio between clusters. Notably, the inflammatory extrathoracic-advanced phenotype (Cluster 2) and acute-markedly reduced lymphocyte phenotype (Cluster 3) had significantly higher SUV ratios than Cluster 1. With a median SUV ratio below 2, Cluster 1 was mostly comprised of subjects with negative PET scans. Conversely, Cluster 2 and 3 both had median SUV ratios ≥2 suggesting more subjects had positive PET scans (odds ratio 6.00 and 6.50, respectively). SUV ratios did not vary between Clusters 2 and 3.

**Figure 5:** Box and whisker plots in **(A)** demonstrate the association between UIC-Sarcoidosis cohort clusters and the SUV_Background_-to-SUV_Max_ ratio (SUV ratio). An SUV ratio of 2 was pre-specified as a cutoff value to indicate increased inflammatory activity on 18FDG-PET/CT (PET-positivity) and is depicted in **(A)** as the dashed black horizontal line. A significant association between clusters and SUV ratio was found by Kruskal-Wallis test (*p* = 0.0052). *Post-hoc* analysis with Dunn's test demonstrated significantly elevated inflammatory activity, denoted with an asterisk (*), in Clusters 2 and 3 compared to Cluster 1 (BH-adjusted *p* = 0.0332 and 0.0136, respectively). No difference (NS) was observed between Cluster 2 and Cluster 3 with regards to inflammatory activity. To assess the probability of PET-positivity based on clusters, a logistic regression model was constructed and the dot plot in **(B)** highlights the odds ratios derived from the model. Cluster 1 was considered the reference given that it demonstrated significantly decreased 18FDG-PET/CT activity compared to the other two clusters. Ultimately, Cluster 2 and Cluster 3 were found to have a 6 and 6.5-fold greater risk of PET positivity (β = 1.7918 and 1.8718 and *p* = 0.0132 and 0.0061; respectively).

As both the inflammatory extrathoracic-advanced phenotype (Cluster 2) and the acute-markedly reduced lymphocyte phenotype (Cluster 3) had high rates of PET avidity, we further investigated the relationship between inflammatory cells and PET positivity in the entire cohort. Receiver operator characteristic (ROC) analysis demonstrating the sensitivity and specificity of absolute neutrophils, absolute lymphocytes, and CD4+ T-cells as predictors of sarcoidosis inflammatory activity on PET scan are shown in Figure 6. Absolute lymphocytes and CD4+ T-cells predict PET positivity with an AUC of 69.20% and 73.42%. There was no difference between their AUC (*p* = 0.36) and both represent strong associations with increased PET avidity and had significantly greater AUC than the absolute neutrophils (*p* = 0.0223 for lymphocytes and *p* = 0.0029 for CD4+ T-cells). Optimal cell count thresholds for the UIC-Sarcoidosis cohort, obtained with “Youden's index,” suggest that absolute lymphocyte counts ≤1.25 kcells/μL and CD4+ T-cell counts ≤524.5 cells/μL are associated with PET scan positivity with median sensitivity of 51.72 and 68.97% and a median specificity of 82.76 and 72.41%, respectively.

**Figure 6:** Receiver operating characteristic (ROC) curves demonstrating the sensitivity and specificity of inflammatory cells as predictors of PET-positivity defined as an SUV ratio > 2. Neutrophils (kcells/μL) demonstrated an area under the curve (AUC) of 45.78% whereas lymphocytes (kcells/μL) and CD4+ T-cells (cells/μL) demonstrated a 69.2 and 73.42% AUC, respectively. No difference was identified between the lymphocyte and CD4+ T-cell AUC utilizing the “bootstrap” method with 1,000 replicates (*p* = 0.36). Both lymphocytes and CD4+ T-cells demonstrated a significantly greater AUC compared to neutrophils (*p* = 0.0223 and 0.0029, respectively). Optimal cell count thresholds obtained with “Youden's index” suggest that lymphocyte counts ≤ 1.25 kcells/μL in the UIC-Sarcoidosis cohort are most indicative of PET-positivity with a median sensitivity of 51.72% (95%CI: 34.48–68.97) and a median specificity of 82.76% (95% CI: 68.97–93.1). Similarly, CD4+ T-cell counts ≤ 524.5 cells/μL were most indicative of PET-positivity with a median sensitivity of 68.97% (95%CI: 51.72–82.76) and a median specificity of 72.41% (95% CI: 55.17–89.66).

To further quantify the inflammatory activity on PET scans, we next assessed TMV and TLG, to compare FDG more stringently between phenotypes (Figure 7). The chronic-quiescent phenotype (Cluster 1) had near normal TMV and TLG values suggesting minimal, if any, FDG avidity and were therefore essentially negative PET scans. This was consistent with the SUV ratio <2 and is therefore not surprising. These values were also significantly lower than the other groups. The inflammatory extrathoracic-advanced cluster (Cluster 2) and the acute-markedly reduced lymphocyte cluster (Cluster 3) had significantly higher TMV and TLG suggesting more sarcoidosis related inflammatory activity (KW-test *p* = 0.01397). PET avidity was further classified into intra and extra-thoracic activity to confirm true extrathoracic involvement in Cluster 2 as suggested by laboratory values. There was no significant difference between clusters in regards to intrathoracic metabolic volume (MV) and lesion glycolysis (LG) (Figures 7C,D, respectively); however, Cluster 2 had significantly higher extrathoracic MV (Figure 7E) and LG (Figure 7F) than both Cluster 1 and Cluster 3 (BH-*adj p* = 0.059 and BH-*adj p* = 0.055, respectively). When comparing the phenotypes identified via cluster analysis with PET avidity, Cluster 1 is consistently quiescent while Cluster 2 and 3 are both hyperinflammatory; Cluster 2 is also confirmed to have more extrathoracic disease.

**Figure 7:** Box and whisker plots demonstrating log_10_ normalized median and interquartile ranges of radiomic measurements performed to assess burden of inflammatory activity in the UIC-Sarcoidosis cohort clusters. **(A,B)** Depict total metabolic volume (TMV) and total lesion glycolysis (TLG). **(C–F)** Depict intrathoracic metabolic volume MV_IT_, intrathoracic lesion glycolysis LG_IT_, extrathoracic metabolic volume MV_ET_, and extrathoracic lesion glycolysis LG_ET_, respectively. Comparisons between clusters were performed with Kruskal-Wallis tests and, if significant (*p* < 0.05), were followed by *post-hoc* analysis with Dunn's test. Dunn's test was considered significant if BH-adjusted *p* < 0.1. Kruskal-Wallis test *p*-values are displayed in their respective panels; brackets above box and whisker plots denote significance of Dunn's test with an asterisk (*). NS, non-significant. Results of significant Dunn's tests: **(A)**- Cluster 1 vs. 2 (BH-adjusted *p* = 0.0237) and Cluster 1 vs. 3 (BH-adjusted *p* = 0.0410); **(B)**- Cluster 1 vs. 2 (BH-adjusted *p* = 0.0170) and Cluster 1 vs. 3 (BH-adjusted *p* = 0.0293); **(E)**- Cluster 1 vs. 2 (BH-adjusted *p* = 0.0096) and Cluster 2 vs. 3 (BH-adjusted *p* = 0.0409); **(F)**- Cluster 1 vs. 2 (BH-adjusted *p* = 0.0058) and Cluster 2 vs. 3 (BH-adjusted *p* = 0.0381).

## Discussion

We have identified phenotypes of sarcoidosis in a diverse tertiary sarcoidosis referral center using unsupervised cluster analysis. We also examined the association between these phenotypes and the extent of sarcoidosis related inflammation. Our unbiased approach yielded 3 distinct clusters, (A) a predominant African American group of treatment naïve subjects with chronic sarcoidosis and minimal inflammatory activity on laboratory and PET scan values; (B) a predominant African American group of subjects with varying disease acuity requiring treatment, with advanced pulmonary parenchymal changes on CT and inflammation more extrathoracically located as evidenced by laboratory and PET scan values; and (C) a predominant Caucasian group of subjects with acute disease requiring treatment, with significant PET avidity that correlates with more significant absolute lymphocyte and CD4+ T-cell reduction. Dissimilarities observed between clusters (summarized in Table 3) attest to the variable immunogenicity and acuity of sarcoidosis. These findings underscore disparities in disease severity associated with race and to a degree, sex, that have previously been described (1). Prior phenotypic studies support the use of cluster analysis as an approach to identify clinical patterns and dissimilarities among large cohorts (16).

**Table 3:** Summary of the most relevant characteristics that comprise the UIC-Sarcoidosis cohort clusters.

**Summary of cluster characteristics**	**Cluster 1**	**Cluster 2**	**Cluster 3**
Race	African American	African American	Caucasian
Sex^(t)^	Female	Female	Male
Disease Acuity	Chronic	Variable	Acute
Lung Parenchyma	Normal	Mixed	Mixed
		(Nodules & Advanced)	(Nodules & Consolidation/GGO)
Treatment	Naïve	Combination Corticosteroid &	Corticosteroid Monotherapy
		Immune modulator	
Markers of Inflammation	Normal	Elevated	Normal
Absolute Lymphocytes (kcells/uL)^(*)^	Normal	Reduced	Reduced
Absolute CD4+ T-cells (cells/uL)^(*)^	Normal	Reduced	Reduced
18FDG-PET/CT	Normal	Positive	Positive

(t) Indicates that a trend toward significance was observed between clusters (Kruskal-Wallis p = 0.0560).

(*) *Reduced peripheral lymphocyte counts and reduced absolute CD4+ T-cell counts within the UIC-Sarcoidosis cohort clusters are defined as median values ≤ 1.5 kcells/uL and ≤ 500 cells/uL, respectively*.

With significantly lower 18-FDG avidity, Cluster 1 identifies subjects with likely inactive sarcoidosis. Conversely, Clusters 2 and 3 are characterized by more subjects with positive PET scans and substantially greater TMV and TLG, consistent with more inflammatory activity and therefore active disease. Using the AUC of the ROC as an integrated measure of test performance, CD4+ T-cell count best predicted increased PET scan activity, though was not statistically superior to the absolute lymphocyte count threshold of 1.25 kcells/μL in our cohort. Notwithstanding, our independent analysis determined that a CD4+ T-cell count of ≤ 524.5 cells/μL is related to PET positivity and note that this was comparable to threshold levels previously utilized to assess major organ involvement in sarcoidosis (7). Despite the need for external validation, we conclude that absolute CD4+ T-cell counts, or absolute lymphocyte counts in lieu of CD4+ T-cell enumeration, may serve as a predictor of sarcoidosis inflammatory activity.

Notably, in our cohort, while the quiescent phenotype was more treatment naïve, all phenotypes had similar rates of corticosteroid use, in combination with other immunomodulators or as monotherapy, and consequently were not considered to significantly influence the degree of lymphocyte reduction across clusters. As sarcoidosis is predominantly a T-helper cell mediated disease, mitigation of inflammation with use of corticosteroids, antimalarials, TNF-α antagonists, among others, has been a mainstay of treatment (49). Phenotype identification has the potential to guide therapy as has been previously shown in successful treatment of patients with sarcoidosis and CD4+ T-cell lymphopenia with the TNF-α antagonist, infliximab (50). Furthermore, use of PET scan has been described as an effective way to assess treatment response (26, 27). Thus, absolute lymphocyte counts and corresponding trends may be considered a useful parameter for monitoring therapy in addition to a surrogate for active inflammation in sarcoidosis.

A further comparison between Clusters 2 and 3 shows both clusters contain subjects with a reduction in the absolute lymphocyte count. However, the degree of reduction was only significant in the Caucasian/acute cluster and further characterized by a corresponding reduction in CD4+ T-cell counts. While we suspect immune dysregulation inherent to sarcoidosis drives peripheral lymphocyte depletion in this cluster, the effect seems to be present primarily in Caucasians, which is consistent with prior gene studies performed on the ACCESS cohort which was notably also predominantly Caucasian (4). Conversely, African Americans belonging to Cluster 3 did not have statistically lower absolute lymphocyte or CD4+ T-cell counts when compared to African Americans in other clusters. However, our cohort was comprised of only a small number of African Americans with acute disease and is a factor that limits full examination of this aspect and should be investigated in subsequent studies. Cluster 2 was characterized by more extrathoracic PET avidity, which is evident in the abnormalities in liver function tests and inflammatory markers. This group also had relatively more normal lymphocyte counts in comparison to Cluster 3, but overall still exhibited decreased absolute lymphocyte and CD4+ T-cell counts. As Cluster 2 was predominantly African American, there were too few Caucasians in this cluster to effectively assess features that distinguish Caucasians in this cluster from Caucasians in other clusters. Nonetheless, our findings suggest that race may influence immunotypes and underscores the importance of health disparities research in sarcoidosis.

Other than differences in lymphocytes, disease chronicity and radiographic findings on CT were also cluster defining features. Subjects in Cluster 1 had more chronic disease and more normal findings on CT, suggesting this cluster represents patients with resolved sarcoidosis. While Cluster 1 was predominantly African American, these findings were consistent when comparing Caucasians across clusters. Additionally, subjects in Cluster 2 had a higher frequency of advanced pulmonary parenchymal disease which may also be reflective of chronic active disease while subjects in Cluster 3 had more acute disease. Taken together these findings imply interdependence between disease chronicity and immunogenicity.

Despite our significant findings, there are several limitations to this study that should be the focus of future works. First, our study was limited by its retrospective design which did not allow full clinical assessment, such as specific organ involvement, at the time of PET scan and precluded the use of predictive tools such as the WASOG organ assessment instrument in the clustering algorithm which may have contributed to improved cluster determination and increased cluster uniformity (13). As with clinical data, acquisition of laboratory data relating to non-CD4+ T-cells was limited by the retrospective design and would have allowed better characterization of each proposed immunotype (7, 51–54). Additionally, although our cohort is representative of the predominantly African American population we serve and strengthened by strict inclusion criteria, sample size and heterogeneity limited our analysis. Consequently, determination of between cluster dissimilarities, particularly in relation to race and disease chronicity, was not possible. Notably, extrathoracic disease assessment across the cohort was limited as FDG uptake on PET scan was considered excretional in the case of the kidneys or artifact in organs such as the heart and brain. Further limitations include lack of standardization of PET scan in terms of optimal protocols for sarcoidosis and lack of follow up PET scan due to radiation risk or insurance coverage.

In summary, we have identified a novel classification scheme using readily available demographic and clinically relevant data to identify three distinct sarcoidosis phenotypes with significant variation in race, disease chronicity, and inflammation. Whether the different immunotypes are reflective of disease acuity, race, comorbid conditions, or prior treatment remains to be resolved and follow-up studies should attempt to assess these differences in more homogeneous cohorts. However, peripheral reductions in lymphocytes, specifically CD4+ T-cells, were significantly related to inflammation identified on 18FDG-PET/CT and therefore sarcoidosis activity. While this finding is significant, a definitive threshold for clinically relevant lymphopenia has not been well-established in sarcoidosis. Though future prospective studies with larger cohorts are warranted, reductions in peripheral lymphocytes may be considered a determinant of sarcoidosis phenotypes and an indicator of active inflammation on 18FDG-PET/CT. Our study opens new doors for research that will help implement new classification criteria for the diagnosis and treatment of sarcoidosis. Multicenter validation studies will help to determine if this classification scheme can be applied broadly as well as clarify the clinical and immunologic implications of these findings.

## Data Availability Statement

The original contributions presented in the study are included in the article/Supplementary Material, further inquiries can be directed to the corresponding author/s.

## Ethics Statement

The studies involving human participants were reviewed and approved by the University of Illinois at Chicago Office for the Protection of Research Subjects. Subjects provided written informed consent prior to participation in this study.

## Author Contributions

NJS, CA, CV, and DRF conceived and designed the study. Subject enrollment was performed by NJS, CA, DRF, RE-I, SA, and BL. Medical record abstraction was performed by CV, CA, RE-I, SA, and YH. Interpretation of imaging studies was performed by CA, CV, and YL. CA, CV, and DRF analyzed the data. CA, CV, RPB, DLP, PWF, and NJS wrote the manuscript. All authors contributed to the article and approved the submitted version.

## Conflict of Interest

The authors declare that the research was conducted in the absence of any commercial or financial relationships that could be construed as a potential conflict of interest.
